The article "SATB1 Overexpression Regulates the Development and Progression in Bladder Cancer through EMT" was retracted in 2024. Reasons: plagiarized data; plagiarized images; overlap with other authors' work; unreliable results or conclusions.

# SATB1 Overexpression Regulates the Development and Progression in Bladder Cancer through EMT

**DOI:** 10.1371/journal.pone.0117518

**Published:** 2015-02-23

**Authors:** Feng Wan, Chao Cheng, Zongwei Wang, Xingyuan Xiao, Hanqing Zeng, Shian Xing, Xuepan Chen, Jin Wang, Sen Li, Youpeng Zhang, Wei Xiang, Zhineng Zhu, Cameron Johnson, Zhaohui Zhu

**Affiliations:** 1 Department of Urology, Union Hospital, Tongji Medical College, Huazhong University of Science and Technology, Wuhan 430022, Hubei, PR China; 2 Department of General Surgery, Union Hospital, Tongji Medical College, Huazhong University of Science and Technology, Wuhan 430022, Hubei, PR China; 3 Department of Urology Massachusetts General Hospital, Harvard Medical School, 55 Fruit St, Warren Building 317, Boston, MA, 02114, United States of America; 4 Central Laboratory of Union Hospital, Tongji Medical College, Huazhong University of Science and Technology, Wuhan 430022, Hubei, PR China; 5 Department of Urology, Wuhan No.1 Hospital, Tongji Medical College, Huazhong University of Science and Technology, Wuhan 430030, Hubei, PR China; 6 Department of Chemistry, Connecticut College, 270 Mohegan Avenue, New London, CT, 06320, United States of America; University of Birmingham, UNITED KINGDOM

## Abstract

The global gene regulator Special AT-rich sequence-binding protein-1 (SATB1) has been reported to induce EMT-like changes and be associated with poor clinical outcome in several cancers. This study aims to evaluate whether SATB1 affects the biological behaviors of bladder transitional cell carcinoma (BTCC) and further elucidate if this effect works through an epithelial-mesenchymal transition (EMT) pathway. The expression of SATB1, E-cadherin (epithelial markers), vimentin (mesenchymal markers) in BTCC tissues and adjacent noncancerous tissues, as well as in two cell lines of bladder cancer were investigated. Whether the SATB1 expression is associated with clinicopathological factors or not was statistically analyzed. Cell invasion and migration, cell cycle, cell proliferation and apoptosis were evaluated in SATB1 knockdown and overexpressed cell lines. Our results showed that the expression of SATB1 was remarkably up-regulated both in BTCC tissues and in bladder cancer cell lines with high potential of metastasis. The results were also associated with EMT markers and poor prognosis of BTCC patients. Moreover, SATB1 induced EMT processes through downregulation of E-cadherin, upregulation of E-cadherin repressors (Snail, Slug and vimentin). SATB1 also promoted cell cycle progression, cell proliferation, cell invasion and cell migration, but did not alter cell survival. In conclusion, our results suggest that SATB1 plays a crucial role in the progression of bladder cancer by regulating genes controlling EMT processes. Further, it may be a novel therapeutic target for aggressive bladder cancers.

## Introduction

Bladder cancer (BC) is one of the most common malignant neoplasms affecting the lining of the urinary bladder, with an estimated 386,300 new cases and 150,200 deaths from the disease worldwide, per year [1]. In China, it has been reported that BC is the most common genitourinary malignancy, and the incidence of this disease has been increased in the last decades [2]. Due to the high local tumor recurrence, further progression and distant metastases, poor clinical outcome has been shown for BC patients, despite the considerable improvements in surgical techniques and adjuvant therapies [3–6]. Meanwhile, the complicated pathways during oncogenesis and the unpredictable biological behavior of cancer are still poorly understood and affected by environmental and genetic factors [7]. Therefore, identification of novel molecular markers which could serve as standard prognostic factors is needed for early diagnosis and for the development of more efficient treatment for BC patients.

It has been generally acknowledged that poor prognosis of malignancies is associated with tumor aggressiveness. This occurs when noninvasive cells become invasive through several metastatic steps, such as the epithelial cells losing polarity and further invading vascular and lymphatic compartments [8]. The epithelial mesenchymal transition (EMT) is the key process which initially occurs during critical phases of embryonic development in which cells lose their epithelial characteristics and cell-cell contacts, and concomitantly acquire migratory and invasive properties of mesenchymal cells [9–11]. Furthermore, similar EMT-like processes might occur during tumor progression in carcinomas and have a promoting role in preventing apoptosis and senescence of tumor cells, contributing to immunosuppression [12]. Loss of E-cadherin expression is a hallmark of the EMT process [9]. Again, in recent studies, transcription factors such as Snail and Slug have been identified as direct repressors of E-cadherin and inducers of EMT, which further elicits complete EMTs at both the morphologic and behavioral levels when overexpressed in epithelial cells[13–15]. In addition, a growing body of evidence suggests that the EMT plays a pivotal role in the initiation and development of metastasis during tumor invasion and progression of bladder cancer *in vivo* and *in vitro* [16–18].

Special AT-rich binding protein 1 (SATB1) is a nuclear matrix attachment region (MAR) DNA-binding protein which acts as a genome organizer and gene regulator through modulating the spatial conformation of chromatin. It also participates in a variety of biologically important processes such as proliferation, differentiation, apoptosis and the reprogramming of expression profiles [19–21]. In recent studies, the upregulation of SATB1 has been found to be correlated with invasion and metastasis of many types of malignances, including gastric cancer, breast cancer, rectal cancer, liver cancer, and prostate cancer. These findings suggest that SATB1 is an independent prognostic factor and a potential therapeutic target in human cancers [21–26]. For instance, Han et al found that SATB1 depletion could reverse the EMT process through down-regulation of E-cadherin repressors such as Snail and SIPI and upregulation of E-cadherin in highly aggressive (MDA-MB-231) cancer cells [21]. Another study reported that chemotherapeutic suppression of miR-448 increases the mRNA levels of SATB1 and promotes the EMT. These findings provide potential novel therapeutic approaches for bladder cancer.

While bladder transitional cell carcinoma (BTCC) is one of the most common sub-types of BC, the current knowledge about the specific mechanism of BTCC invasion and metastasis is still limited. In one recent study, Bin Han et al found that SATB1 was overexpressed in human bladder cancer and associated with tumor grade and stage. In addition, they also found that SATB1 depletion decreased cell proliferation and increased cell apoptosis in 5637 and T24 cells [27]. However, how the expression of SATB1 affects the biologic behavior of BTCC and whether SATB1 induces the EMT in bladder cancer is still unexplored. In this study, we evaluated the expression of SATB1 in BTCC specimens and bladder cancer cell lines though immunohistochemical staining, Real-Time RT-PCR assays and western blotting analysis and found that its expression is correlated with clinically pathological characteristics. In established human bladder cancer cell lines, we further demonstrated that overexpressed or silenced SATB1 regulated the cell migration, invasion and proliferation, along with the cell cycle.

## Materials and Methods

### Materials

Primary bladder cancer specimens and matched non-cancerous tissues were obtained from 126 patients (mean age 65.2 years, range 45–78) diagnosed with bladder cancer who underwent surgical resection for immunohistochemical assays at Union Hospital in the Department of Urology (Wuhan, China) between April 2007 and October 2012. Parts of tissue samples were fixed in formalin and embedded in paraffin. All of the patients did not receive preoperative treatment, such as chemotherapy or radiation. All the participants provided their written informed consent to participate in this study, and the study was approved by the Ethics Committee of Union Hospital, Tongji Medical College, Huazhong University of Science and Technology (HUST). Clinical and pathologic information was obtained from a retrospective review of well-documented medical records. Tumors were classified histologically as non-muscle-invasive bladder cancer (NMIBC) (stage pTa) or muscle invasive bladder cancer (MIBC) (stage pT3) according to tumor-nodes-metastasis (TNM) classification for the stage [28]. Grade was assigned according to the World Health Organization’s classification of tumors of the Urinary System and Male Genital Organs (2004) [28]. All deaths were attributable to bladder cancer. Patient characteristics are detailed in Table 1. Human bladder cancer cell lines BIU-87 and T24 were maintained in our laboratory (Central Laboratory of Union Hospital, Tongji Medical College, HUST, Wuhan, China). BIU-87 cells were derived from a grade II, non-muscle-invasive (pT1) human BTCC of the urinary bladder. T24 cells, which are poorly differentiated and possess a higher potential of metastasis and display a typical fibroblastic morphology microscopically were derived from a grade III bladder carcinoma [29]. The cells were cultured in RPMI-1640 medium supplemented with 10% fetal bovine serum and 100μg/ml penicillin-streptomycin (Gibco, Carlsbad, CA, USA), and incubated with a humidified atmosphere of 95% air and 5% CO_2_ at 37°C.

**Table 1:** Relationships between SATB1 mRNA expression and clinicopathological characteristics.

Characteristics	SATB1 mRNA expression			P-value
	n	High(n = 71)	Low (= 55)	
Age				0.034
≥55	57	38	19	
<55	69	33	36	
Gender				0.143
Male	83	45	38	
Female	43	26	17	
Tumor differentiation				0.111
Well(G1)	58	32	26	
Moderately and poorly(G2–G3)	68	39	29	
Depth of invasion				0.000
T1+T2	59	23	36	
T3+T4	67	48	19	
TNM stage				0.015
I+II	49	21	28	
III+IV	77	50	27	
Lymph node metastasis				0.013
Absent	34	13	21	
Present	92	58	34	
Distant metastasis				0.012
Absent	102	52	50	
Present	24	19	5	

### Immunohistochemical staining analysis

Protein expression was determined by immunohistochemical staining for SATB1, E-caderin and vimentin, with the streptavidin biotin-peroxidase complex method using SABC kits (Boster Ltd., Wuhan, China) according to the manufacturer’s protocol. Briefly, tissue specimens were fixed in 10% neutral buffered formalin, dehydrated and embedded in paraffin. Then, the sections were deparaffinized and rehydrated. Hydrogen peroxide was applied to block endogenous peroxide activity for 10 min. After antigen retrieval using a microwave, the sections were treated with 10% normal goat serum for 10 min at room temperature to reduce the nonspecific binding capacity. The sections were then incubated with rabbit polyclonal antibody SATB1, E-caderin and vimentin (Abcam Inc., Cambridge, MA, USA) at the dilution of 1:70. These were left in a humidified chamber overnight at 4°C. After washing three times with phosphate-buffered saline (PBS) for 5 min each time, the sections were incubated with secondary antibody for 40 min and then with Streptavidin biotin-peroxidase complex for 40 min at 37°C. After rinsing, diaminobenzidine (DAB; Abcam Inc., Cambridge, MA, USA) was used as chromogen and the sections were counterstained with hematoxylin. Samples incubated with PBS instead of the primary antibody served as negative controls. SATB1staining in nuclear was defined as detectable immunoreactions and E-caderin and vimentin staining in plasmalemma or cytoplasm was defined as detectable immunoreactions. The positive staining was scored based on the intensity and percentage of cells with SATB1 nuclear staining. According to the predominant intensity, staining intensity was denoted on the following scale: score 0, negative nuclear staining for all tumor cells; score 1, weak nuclear staining; score 2, moderate nuclear staining; score 3, strong nuclear staining. According to the percentage of positively stained cells, the score of staining density was given as follows: 0, less than 5%; 1, 5 to 25%; 2, 25 to 50%; 3, more than 50%. The final score was calculated by adding the two above scores. Scores of 0–2 were defined as low expression scores, and 3–6 were defined as high scores.

### RNA extraction and quantitative real-time PCR assays

Total RNA was extracted and purified from each tissue sample and cell lines using the Trizol reagent (Invitrogen Corporation, Carlsbad, CA, USA) according to the manufacturer’s instructions. Reverse transcription was performed using the reverse transcription kit (Takara Biotechnology Dalian, China) with the following conditions: reverse transcription at 37°C for 25 min, followed by incubation at 85°C for 5 sec in 20 μl of reaction volume. Then the cDNA was prepared and used as a template for quantitative real-time polymerase chain reaction (PT-PCR) performed on an ABI StepOnePlus Real-Time PCR System (Applied Biosystems Inc., Foster City, CA) using the SYBR Green Real-time PCR Master Mix (Takara Clontech, Kyoto, Japan). This was done with the following conditions: denaturation at 95°C for 30 seconds, followed by 40 cycles of amplification (95°C for 5 seconds, 60°C for 30 seconds). Primers were designed using NCBI Primer-BLAST as follows: SATB1 (forward, 5′-GTGGAAGCCTTGGGAATCC-3′; reverse, 5′-CTGACAGCTCTTCTTCTAGTT-3′), E-cadherin (forward, 5′-CTG GACGCTCGGCCTGAAGT-3′; reverse, 5′-GGGTCAGTATCAGCCGCTTT-3′), Vimentin (forward, 5′-ACAGGCTTTAG CGAGTTATT-3′; reverse, 5′-GGGCTCCTAGCGGTTTAG-3′), Twist (forward, 5′- CAGCGCACCCAGTCGCTGAA-3′; reverse, 5′-CCAGGCCCCCTCCATCCTCC-3′), Snail (forward, 5′-ATCCGAAGCCACACGCTGCC-3′; reverse, 5′-CACGGCTGCAGTGGGGACAG-3′), Slug (forward, 5′-CGCTCCTTCCTGGTCAAGA-3′; reverse, 5′-TTGCGTCACTCAGTGTGC-3′), ZEB1:(forward, 5′-TGCTCCCTGTGCAGTTACACCTT-3′; reverse, 5′-CCAGACTGCGTCACATGTCTTTGA-3′), ZEB2: (forward, 5′-ATACCGCGGTGCCATCCTTGTACAGTGGTT-3′; reverse, 5′-GCGCTGCAGAGTAATTGGAAAAAAACAAA-3′), GAPDH (forward, 5′-TCGGAGTCAACGGATTTGGTCGT-3′; reverse, 5′-TGCCATGGGTGGAATCATATTGGA-3′). The primers were designed to be intron-spanning. The cycle threshold (CT) values were standardized to CT values of GAPDH. The relative levels of individual mRNA in each sample transcript compared to control GAPDH were calculated using the 2^-ΔΔCt^ method.

### Western blotting analysis

Total protein was extracted from each tissue sample and cell line using RIPA Buffer (Sigma, St Louis, MO, USA) according to the manufacturer’s instructions. Protein concentrations were determined with a BCA Protein Assay Kit (Boster Ltd., Wuhan, China). Equal amounts of harvested protein samples were resolved on a 10% sodium dodecyl sulfate-polyacrylamide gel electrophoresis (SDS-PAGE) (Bio-Rad, Hercules, CA) and transferred to PVDF membranes (Millipore Corporation, Billerica, MA, USA) followed by blocking with TBST buffer composed of 50 mM Tris (pH 7.6), 150 mM NaCl, and 0.05% Tween supplemented with 5% fat-free milk at 4°C for 2 hour. The blotted membranes were incubated overnight at 4°C with rabbit polyclonal antibody SATB1, E-cadherin, vimentin (Abcam Inc., Cambridge, CA, USA) (1:800), ZEB1, ZEB2, Snail and Slug (Santa Cruz Biotechnology Inc., Santa Cruz, CA, USA) (1:500). We used GAPDH (Boster Ltd., Wuhan, China) as a loading control. Antibody binding was detected using peroxidase-conjugated secondary antibodies (Boster Ltd., Wuhan, China) for another 2 h at room temperature according to the manufacturer’s instructions. The immunoreactive bands were visualized by enhanced Western blotting detection system ECL (Pierce Biotechnology, Rockford, IL, USA) and the intensity of the detected bands was analyzed using an Image J program.

### SATB1-knockdown cells

One previously validated shRNA was used [21]. The sequence of the shRNA was as follows: 5’-GGATTTGGAAGAGAGTGTC-3’. The shRNA was synthesized and cloned into the pGenesil2 vector (GenePharma Co., Ltd. Shanghai, China) and then transfected into 50%-confluent T24 cell line together with a pGenesil2 control vector using Lipofectamine 2000 Reagent (Invitrogen) according to the manufacturer’s instruction. Pooled populations of knockdown cells were obtained after two weeks of drug selection with 400μg/ml G418, following incubation for 24 h. Then the stable RNA-interference-mediated SATB1-knockdown cell lines were designated as pGenesil2-SATB1-shRNA and were further cultured for the subsequent experiments. T24 cells treated with pGenesil2-scrambled-shRNA (5’-TTCTCCGAACGTGTCACGT-3’) which does not target any specific gene were used as the control groups.

### SATB1-overexpressing cells

The human full-length SATB1 cDNA was cloned into the pcDNA3.1 expression vector purchased from GenePharma Co., Ltd. (Shanghai, China). After being confirmed by DNA sequencing, the pcDNA3.1-SATB1 expression vector and pcDNA3.1 control vector were transfected into 50%-confluent BIU-87 cells using Lipofectamine 2000 respectively (Invitrogen). After transfection, stable cell lines were selected after incubation with 600μg/ml of G418 in RPMI-1640 medium supplemented with 10% fetal calf serum for two weeks. These were then cultured for the subsequent experiments. The SATB1-overexpressing BIU cells were established and the SATB1 expression levels shown by these cells were confirmed using Real-Time RT-PCR analysis. Nontransfected BIU-87 cells were used as the control groups.

### Immunofluorescence analysis

To determine protein cellular localization for SATB1 and E-cadherin, immunofluorescence was performed using an A1Si laser-scanning confocal microscope. Briefly, BIU-87 and T24 cells transfected with pcDNA3.1-SATB1 and pGenesil2-SATB1-shRNA expression vectors were seeded onto glass coverslips and placed in 24-well plates. Cells were fixed with 4% paraformaldehyde for 30 min at 37°C after incubation for 3 days, and then washed with PBS twice for 10 minutes each. The fixed cells were permeabilized with 0.3% Triton- X 100 for 15 min, blocked in 10% goat serum for 1h, and then washed with PBS twice for 10 minutes each. Then the cells were incubated with primary antibody as follows: rabbit polyclonal antibody SATB1, and E-cadherin(Abcam Inc., Cambridge, CA, USA) (1:50) at 4°C overnight followed by detection with Cy5-conjugated secondary antibodies and FITC-labelled phalloidin (5μg/ml)(sigma) for 1 hour at room temperature in the dark. DAPI was subsequently used to stain nuclei. Images were collected using a Nikon A1Si laser-scanning confocal microscope (Nikon, Japan).

### Cell invasion and migration assays in vitro

BIU and T24cells transfected with pcDNA3.1-SATB1 plasmids, pGenesil2 vector containing SATB1-specific shRNA as well as the negative control vector were added to the upper compartment of the transwell plates with 6.5 mm poly-carbonate filters and 8.0μm pore size (Corning Costar, MD, USA). This was done in 100μL of serum-free media and 500μL of RPMI-1640 containing 10% FBS. For cell invasion assays, the transwell filter inserts were coated with 50μL Matrigel(BD Biosciences, NJ, USA). After incubation for 12h at 37°C, 5% CO_2_ atmosphere, the tumor cells that penetrated the bottom of the insert membrane were fixed in 4% paraformaldehyde and stained with Crystal Violet (Boster Ltd., Wuhan, China) according to the manufacturer’s protocol. Then the invasive stained cells were counted under a light microscope in 10 randomly selected fields at 200 × magnification. For cell migration assays, transfected cells were seeded in upper chambers without coated Matrigel. After incubation for 12h at 37°C, 5% CO_2_ atmosphere, the migrated cells on the undersides of filter membrane were fixed and stained with Crystal Violet and then counted and analyzed as described above. Three replicate wells were tested per assay, and each experiment was performed in triplicate. Spectrophotometer was used to measure the optical density at 560 nm, and the ability of cell invasion was calculated using the percentage of the cells that penetrated the Matrigel-coated filters.

### Cell cycle and proliferation analysis

To validate the effects of SATB1 on the cell cycle, flow cytometry was used to analysis the percentage of cells in each cell cycle phase after cell staining with propidium iodide (PI) (Keygentec, China) according to the manufacture’s protocol. In brief, BIU and T24 cells were resuspended in ice-cold PBS and fixed with 70% ethanol on ice. Then the fixed wells were stained with PI solution for 30 min and analyzed by flow cytometry.

CCK-8 cell proliferation assay (CCK-8 kit; Boster Ltd., Wuhan, China) was used to detect the cell growth rates according to the manufacturer’s instructions. In brief, the established SATB1-knockdown T24 cells and SATB1-overexpressing BIU-87 cells at 4×10^3^ per well were seeded in flat-bottomed 96-well plates and incubated for 48 h at 37°C, in a 5% CO_2_ atmosphere. For quantitation of cell viability, cells were incubated with a CCK-8 solution (10μl/ well) for 1.5 h at 37°C. Then the absorbance values of tumor cells were measured at 450 nm at indicated time points using a microplate reader (Bio-Rad, Tokyo, Japan). Three replicate wells were tested per assay, and each experiment was performed in triplicate.

### Apoptosis assay

To detect the effects of SATB1 on cell apoptosis, flow cytometry was performed to analyze the apoptotics rate using Annexin V-FITC Apoptosis Detection Kit (Keygentec, China) according to the manufacture’s protocol. In brief, BIU and T24 cells transfected with pcDNA3.1-SATB1 plasmids and pGenesil2 vector containing SATB1-specific shRNA as well as negative control vector were plated in 6-well plates and cultured for 24 hours. Then the cells (1x10^6^) were stained with Annexin-V and PI and the apoptotic cells were determined by the Annexin V-FITC apoptosis detection kit and assessed using a FACSCalibur instrument.

### Statistical analysis

The data are presented as mean ± standard error of the mean (SEM). Three replicate wells were tested per assay, and each experiment was performed in triplicate. Statistical comparisons between groups were determined by the student’s *t*-test. Cross-table analysis was performed using Pearson’s chi-squared (χ^2^) test or Fisher’s exact test to analyze the significance of correlations between SATB1 expression and clinicopathological features of bladder cancer. Kaplan—Meier plots were used to estimate the prognostic relevance of SATB1 in a univariate analysis. Multivariate analysis was performed using a COX proportional hazards test. All data were analyzed using SPSS 16.0 (SPSS Inc., Chicago, IL, USA). All statistical tests were two-tailed and statistical significance was assumed for p < 0.05.

## Results

### SATB1 is up-regulated in human BTCC tissues and bladder cancer cell line with high metastatic potential

To investigate whether the abnormal expression of SATB1 is related to bladder cancer development and progression and also involved in regulating EMT in human bladder cancer, immunohistochemistry, real-time RT-PCR and western blotting analyses were initially performed to identify the expression of SATB1. Further they were used to analyze E-cadherin and vimentin in 126 tissue samples of human bladder cancer, corresponding to adjacent normal tissues and bladder cancer cell lines respectively. The expression levels of SATB1 and vimentin were found to be significantly up-regulated at mRNA and protein levels in NMIBC and MIBC tissues compared with those in corresponding adjacent nonneoplastic specimens (Fig. 1A and C; *P < 0.05;**P < 0.001). We also found that there were remarkable changes in the expression levels of SATB1 and vimentin between NMIBC and MIBC tissues, which revealed that MIBC tissues showed higher levels of SATB1 and vimentin than that in NMIBC tissues (Fig. 1A and C; *P < 0.05). The expression levels of SATB1 RNA and protein were significantly higher in metastatic tumor cell line (T24) than that in non-metastatic tumor cell line (BIU-87) (Fig. 1A and C; **P < 0.001), suggesting SATB1 expression was associated with aggressive tumor phenotypes. Furthermore, the expression of vimentin was strikingly upregulated at RNA and protein levels in T24 cell line compared with those in BIU-87 cell lines (Fig. 1A and C; *P < 0.05). Conversely, the E-cadherin expression was markedly low or lost at mRNA and protein levels in NMIBC tissues, MIBC tissues and high metastatic tumor cell line T24 but significantly high in corresponding adjacent non-neoplastic specimens and BIU-87cell line (Fig. 1A and C; *P < 0.05, **P < 0.001). Similar results were obtained by immunohistochemistry staining analysis for detecting SATB1, E-cadherin and vimentin, which showed that SATB1 was predominantly localized in the nuclei of the bladder cancer tissue, with low immunoreactivity in normal bladder tissues (Fig. 1B). However, vimentin was found to be predominantly stained in plasmalemma of bladder cancer tissues, with a loss of or low of E-cadherin staining (Fig. 1B). Among primary bladder cancer patients with positive SATB1 expression displayed lost or low E-cadherin expression but high vimentin expression. In contrast, SATB1-negative patients exhibited strong E-cadherin staining but a light staining of vimentin (Fig. 1D), which suggests a strong positive correlation between SATB1 and EMT markers in BTCC.

**Fig 1:** SATB1 is upregulated in human bladder carcinoma tissues and bladder carcinoma cell lines with high metastatic potential. Expressions of mRNA levels of SATB1, E-cadherin and vimentin in human bladder carcinoma tissues and two bladder carcinoma cell lines were assessed by quantitative RT-PCR (A; *P < 0.05, **P < 0.001). IHC staining of human bladder carcinoma tissues and corresponding adjacent non-cancerous tissues for SATB1, E-cadherin and vimentin was performed. SATB1 staining was observed in the nuclei of bladder cancer cells, vimentin was found to be predominantly stained in plasmalemma of bladder cancer cells, but E-cadherin staining was observed mainly in plasmalemma of non-cancerous bladder cells (B); Bladder cancer samples with SATB1-positive were stained with vimentin but not E-cadherin. However, tumor samples with SATB1-negative were stained with E-cadherin but not vimentin (D). The original magnification was ×400x (B and D). Protein levels of SATB1, E-cadherin and vimentin were examined by western blot (C). Error bars indicate s.e.m., n = 3 experiments.

### Overexpression of SATB1 is associated with clinicopathological parameters and correlates with poor prognosis

The relationships between SATB1mRNA expression and clinicopathological factors were investigated. As shown in Table 1, high expression of SATB1 was significantly associated with age (≥55 vs. <55, p = 0.034), primary tumor depth of invasion (T1 + T2 vs. T3 + T4, P<0.001), TNM stage (stages I + II vs. stages III + IV, P = 0.015), presence of lymph node metastasis (P = 0.013) and presence of distant metastasis (P = 0.012). However, no significant differences were detected between high SATB1 expression and either gender (male vs. female, P = 0.143) or tumor differentiation (G1 vs. G2+G3, P = 0.111). Kaplan-Meier analysis was performed to determine the prognostic significance of SATB1. As shown in Fig. 2, the analysis revealed a correlation between higher SATB1expression levels and shorter overall survival times (P <0.001). Furthermore, multivariable Cox regression analysis confirmed that SATB1 expression is a significant and independent prognostic factor for human bladder transitional cell carcinoma after adjusting for the other factors as shown in Table 2 (P = 0.005).

**Fig 2:** Kaplan-Meier estimates of survival according to SATB1 expression in patients with bladder cancer. The 5-year overall survival rate in patients with high SATB1 expression was significantly worse than those with low SATB1 expression (P<0.001; log-rank test).

**Table 2:** Multivariate analysis for survival by the Cox proportional hazard regression model.

		Multivariate analysis	
Variables	Relative risk	95% CI	P-value
SATB1 expression^a^	0.549	0.362–0.834	0.005
Age^b^	1.019	0.704–1.474	0.921
Gender^c^	1.142	0.771–1.691	0.509
Tumor differentiation^d^	1.227	0.849–1.771	0.276
Depth of invasion^e^	1.364	0.905–2.055	0.138
TNM stage^f^	0.936	0.645–1.360	0.730
Lymph node metastasis^g^	1.149	0.783–1.687	0.478
Distant metastasis^g^	0.824	0.520–1.304	0.408

CI, confidence interval;

^a^high vs. low;

^b^≥55 vs. <55;

^c^male vs. female;

^d^G1 vs. G2–G3;

^e^T1+T2 vs. T3+T4;

^f^I+II vs. III+IV;

^g^absent vs. present.

### Ectopic expression of SABT1 induces EMT in an established human cancer cell line, increasing their invasive capability

Previous studies have linked SATB1expression with epithelial-mesenchymal transition (EMT) [21,24]. To test whether ectopic expression of SATB1 could induce EMT in non-metastatic tumor cells, the human bladder cancer cell line (BIU-87) with very low SATB1 expression was transfected with pcDNA3.1-SATB1 expression plasmids to establish a stable SATB1-overexpressing cell line as described in Material and Methods. The results of real-time RT-PCR and western blotting showed that SATB1 mRNA and protein levels of transfected group significantly increased compared to the nontransfected group and the control vector-transfected group (Fig. 3A; **P < 0.001). However, there were no remarkable changes in the expression of SATB1 in the control vector-transfected group and nontransfected group (P>0.05). Similar results could be obtained by immunofluorescence analysis for detecting SATB1 (Fig. 3C). Interestingly, we found that transfection of BIU-87 cells caused a significant increase of Snail and Slug (mRNA and protein) and a concomitant induction of vimentin (mRNA and protein). The mRNA levels of E-cadherin expression were decreased after transfection of pcDNA3.1-SATB1 expression plasmids (Fig. 4A; P < 0.05). However, there were no remarkable changes in the expression of E-cadherin protein between the control vector and the pcDNA3.1SATB1 group (Fig. 4B; P > 0.05). There was only a trend for reduction in E-cadherin protein expression, and the inhibited effect was not as pronounced because the inhibition might be post-translational.

**Fig 3:** The SATB1-overexpressing cells and SATB1-knockdown cells are established. The SATB1 expression of BIU-87 cells and T24 cells transfected with pcDNA3.1-SATB1 and pGenesil2-SATB1-shRNA were examined by qRT-PCR and western blot (A and B; **P < 0.001). Non-transfected BIU-87 cells were used as control group. T24 cells treated with pGenesil2 control vector which does not target any specific gene were used as the control groups. Immunofluorescence analysis was performed to detect the SATB1staining in each cell groups. Immunofluorescence images at 200×magnification (C and D). Error bars indicate s.e.m., n = 3 experiments.

**Fig 4:** Ectopic expression of SABT1 induces EMT and knockdown of SATB1 reverses EMT in established human cancer cell lines. The expression of Snail and Slug, two inhibitors of E-cadherin, and the mesenchymal marker vimentin were upregulated after SATB1 expression was enhanced (A; **P<0.001). The mRNA levels of E-cadherin expression were decreased after transfection of pcDNA3.1-SATB1 expression plasmids (A; P < 0.05). There was a trend for reduction in E-cadherin protein expression in BIU-87 cells with enhanced SATB1 expression (B; P>0.05). After SATB1 expression was silenced with SATB1 shRNA in T24 cells, the expression of Snail, Slug and mesenchymal markers vimentin was downregulated. The expression of epithelial marker, E-cadherin, was upregulated compared to nontransfected cells and control vector-transfected cells (C and D; *P<0.05;**P<0.001). There were no remarkable changes in the expressions of ZEB1, ZEB2 and Twist, other known inhibitors of E-cadherin, in BIU-87 with enhanced SATB1 expression and T24 cells with reduced SATB1 expression, respectively.

However, there were no remarkable changes in the expression of ZEB1, ZEB2 and Twist, which known as other inhibitors of E-cadherin, in the three cell groups (P>0.05). Furthermore, BIU-87 cells treated with pcDNA3.1-SATB1 expression plasmids exhibited a marked change in morphology, from a cobblestone-shaped morphology to a spindle-shaped morphology (Fig. 5A and C), which is a classical marker of EMT induction. In addition, the E-cadherin was reduced on the plasma membrane in the established pcDAN3.1-SATB1 BIU-87 cells (Fig. 5E). In addition, we found that treatment of pcDNA3.1-SATB1 resulted in a significant increase in migration and invasive capability (Fig. 6A and C). According to morphologic criteria and biochemical and biological behavior, it was showed that BIU-87 cells had undergone a developmental switch from an epithelial to a mesenchymal cell phenotype (Fig. 5A and C). These results indicate that high-level expression of SATB1 is sufficient to induce EMT, maintain aggressive fibroblastic morphology and promote invasion and migration of BIU cells.

**Fig 5:** SATB1 induces EMT-like changes in bladder cancer cells. BIU-87 cells with enhanced SATB1 expression exhibited a marked change, from a cobblestone-shaped morphology to a spindle-shaped morphology (A and C), a classical marker of EMT. T24 cells with reduced SATB1 expression showed a major cell morphological change, from a spindle-like fibroblastic morphology to a cobble-stone-like morphology (B and D), consistent with the cells undergoing MET. The images of cell morphological changes were collected using an inverted microscope at 200×magnification(A and B) and A1Si laser-scanning confocal microscope at 400×magnification (C and D; scale bar = 20 μm) in each group cells. Photographs of representative cells are shown (C and D). The E-cadherin was reduced on the plasma membrane in the established pcDAN3.1-SATB1 BIU-87 cells, but was founded to be enriched in SATB1-shRNA T24 cells (E and F).

**Fig 6:** Cell invasion and migration capability *in vitro* were detected by transwell invasion and migration assay. The cells invading the lower chamber were stained with crystal violet, photographed, and then extracted with 10% acetic acid. Representative images of cell migrations to the bottom chamber are shown (A and B). BIU-87 cells with enhanced SATB1 expression exhibited increased invasiveness and T24 cells with reduced SATB1 expression showed reduced invasiveness, when compared to control groups (C and D;*P < 0.05). Error bars indicate s.e.m., n = 3 experiments.

### Knockdown of SATB1 reverses epithelial-mesenchymal transition (EMT) in established human cancer cell lines, reducing their invasive capability

In an experimental model which used an established breast tumor cell line, MDA-MB-231 and liver tumor cell line, SK-HEP-1 with a highly aggressive potential, researchers found that SATB1 depletion could reverse the epithelial-mesenchymal transition (EMT) process. This is due to downregulation of Snail, SIP1 (ZEB2) and Slug, and upregulation of E-cadherin [21,24]. We therefore investigated whether SATB1 knockdown could affect marker expression in a way consistent with EMT or MET induction in a SATB1 high-expressing cancer cell line (T24). This line presented a high metastatic potential and displayed a typical fibroblastic morphology. Stable RNA-interference-mediated SATB1-knockdown cell line T24 was established as described in Material and Methods. After transfection with pGenesil2-SATB1-shRNA, the expression of SATB1 protein in SATB-shRNA cells became hardly detectable by immunoblotting and its mRNA levels were significantly reduced (Fig. 3B; **P < 0.001), while the expression of SATB1 in control vector-transfected cells remained unaltered (P >0.05). These differences were confirmed by immunofluorescence analysis (Fig. 3D). Consistent with previous studies, we observed that low-level SATB1expression is associated with a significant increase of E-cadherin mRNA and protein and reduced mRNA and protein production for Snail and Slug (Fig. 4C and D; *P < 0.05; **P < 0.001) in the established SATB1-shRNA T24 cells. However, there were no remarkable changes in the expression of ZEB1 and ZEB2 in the T24 cells before and after transfection with pGenesil2-SATB1-shRNA (Fig. 4C and D; P>0.05). In addition, we observed major cell morphological changes, from a spindle-like fibroblastic morphology to a cobble-stone-like morphology (Fig. 5B and D). Furthermore, the E-cadherin was found to be increased on the plasma membrane in the established SATB1-shRNA T24 cells (Fig. 5F). Cell invasion and migration assays showed that the cells transfected with SATB1-shRNA exhibited reduced invasive and migration activity compared to control groups *in vitro* (Fig. 6B and D; *P<0.05). Based on morphologic criteria as well as biochemical and biological behavior, we concluded that SATB1knowdown could reverse EMT and inhibit invasive and migratory capacity, suggesting that SATB1 may exert a crucial role in tumor progression.

### SATB1 promotes cell cycle entry leading to proliferation, but does not alter cell survival

To define the effects of SATB1 on the growth of bladder cancer cells, CCK-8 cell proliferation assays and flow cytometric analysis were performed to evaluate the cell proliferation and cell cycle. After SATB1 expression was enhanced with pcDNA3.1-SATB1 plasmid, the ratio of cells in G0/G1 phase decreased, and the ratio of cells entering S phase increased significantly compared to the control group (Fig. 7A; *P < 0.05). However, there was no significant difference in apoptosis rate between groups (Fig. 7B; P >0.05). Furthermore, BIU-87 cells exhibited a greater proliferative capacity after stable transfection with pcDNA3.1-SATB1 than control group (Fig. 8; *P < 0.05, **P < 0.001). On the contrary, the cell cycle progression was arrested in G0/G1 phase, and the ratio of cells entering S phase was reduced significantly in T24 cells treated with pGenesil2-SATB1-shRNA (Fig. 7A; *P < 0.05). Meanwhile, the proliferation of cells was significantly inhibited in SATB1-knockdown cells compared to control group (Fig. 8, *P < 0.05; **P < 0.001). Nevertheless, the apoptotic rate didn’t increase in SATB1-knockdown cells (Fig. 7B; P >0.05), which was not consistent with the previous studies [27]. On the basis of these findings, our results suggested that SATB1 promotes cell cycle entry leading to proliferation, but does not alter cell survival in bladder cancer cells *in vitro*.

**Fig 7:** Effects of SATB1 on cell cycle progression and apoptosis of BIU-87 and T24 cells *in vitro*. The cell population at each stage of the cell cycle and apoptosis were analyzed by flow cytometry. After SATB1 expression was enhanced with pcDNA3.1-SATB1 plasmid in BIU-87 cells, the ratio of cells in G0/G1 phase decreased, and the ratio of cells entering S phase increased significantly compared to nontransfected cells and control cells (A; *P < 0.05). After SATB1 expression was silenced with SATB1 shRNA in T24 cells, the cell cycle progression was arrested in G0/G1 phase, and the ratio of cells entering S phase was reduced significantly compared to nontransfected cells and control cells (A; *P < 0.05).There were no changes in the apoptosis rate in SATB1-overexpressing BIU-87 cells and in SATB1-lowexpressing T24 cells (B; P > 0.05).

**Fig 8:** Cell proliferation rates were measured by CCK-8 cell proliferation assay. Absorbance at 450 nm was determined at the indicated time points and 630 nm was the reference wavelength (*P < 0.05, **P < 0.001), Error bars indicate s.e.m., n = 3 experiments.

## Discussion

Metastasis of tumor cells to distant organs is the late step in solid tumor progression and the primary cause of death in cancer patients [30,31]. In addition to being essential for embryonic development, EMT is essential in cancer progression, tumor invasion and metastasis through down-regulation of E-cadherin [9,32,33]. EMT is characterized by the loss of intercellular adhesion (E-cadherin), the upregulation of mesenchymal markers (vimentin), and the acquisition of a fibroblast-like motile and invasive phenotype based on experiments *in vitro* [9,34]. Previous studies have indicated that several regulative factors, such as Tβ4, microRNA200, TGF-β1, were involved in the EMT process as direct inducers. SATB1, a cell type-specific nuclear matrix attachment region (MAR) DNA-binding protein, was identified as an additional EMT regulator. It was also found to be overexpressed in the highly invasive and mesenchymal-like breast cancer MDA-MB-231 cells as compared to non-invasive epithelial-like breast cancer MCF7 cells [21]. An accumulating body of evidence indicates that aberrant SATB1expression plays a crucial role in facilitating tumor invasion and metastasis in a large panel of human malignant tumor cells, such as breast tumor cells, liver tumor cells and might contribute to tumor development and progression [21,24]. Mechanisms underlying the global regulatory role for SATB1 during metastasis are based on tethering hundreds of gene loci onto its regulatory network, and by assembling them with chromatin modifying and transcription factors. In this study, we showed that the expression of SATB1 was significantly increased at both mRNA and protein levels in human bladder cancer tissues and in highly metastatic bladder cancer T24 cells than that in corresponding normal tissues and nonmetastatic bladder cancer BIU-87 cells respectively, which was consistent with a previous study[27]. The results mentioned above were confirmed by immunohistochemical analysis for tissue sections and immunofluorescence staining for bladder tumor cells. Moreover, patients with high SATB1 expression displayed strong expression of vimentin but low or lost E-cadherin expression, which was consistent with the results which loss of E-cadherin was known as a pivotal event for EMT[35]. The results suggest there are potentially certain correlations between SATB1 expression and EMT markers in bladder cancer specimens, which show that SATB1 overexpression positively correlate with vimentin expression but inversely with E-cadherin. Consequently, our findings support the emerging links between SATB1 expression and the EMT process.

Han et al revealed that RNA-interference-mediated knockdown of SATB1 reverses the EMT process through downregulation of E-cadherin transcription repressors such as Snail and SIPI and also through upregulation of E-cadherin in highly aggressive (MDA-MB-231) cancer cells [21,24]. To address the precise mechanism(s) for SATB1-induced EMT-like phenotypic changes in cancer cells, researchers established several experimental cell models, finding that overexpression of SATB1 could induce EMT in non-aggressive tumor cells, while SATB1 depletion could reverse EMT in aggressive tumor cells by regulating Snail, Slug and E-cadherin *in vitro*[24]. To confirm whether ectopic expression of SATB1 is sufficient to induce EMT-like changes in bladder cancer cells, we established a SATB1-overexpressing cell line using non-invasive bladder cancer cells (BIU-87). After the SATB1 expression was enhanced, BIU-87 cells displayed typical spindle-shaped fibroblast-like morphology and the expression of Snail, Slug and vimentin were significantly up-regulated, which was in accordance with the phenotypic EMT-like changes. Inversely, the SATB1-knockdown expressing cells established used highly invasive bladder cancer cells (T24) showed cobblestone epithelial morphology instead of the usual spindle-like cell morphology. Moreover, downregulation of repressors of E-cadherin such as Snail and Slug and mesenchymal markers (vimentin) and upregulation of E-cadherin indicate that the cells underwent mesenchymal-epithelial transition (MET). To determine whether the EMT-like or MET-like changes observed in the two established cells after enhance or inhibition of SATB1 were due to the up-regulation or down-regulation of Snail and Slug or other known inhibitors of E-cadherin, we also detected the expression of ZEB1, ZEB2 and Twist [36–39]. However, there were no obvious differences in the expression of ZEB1, ZEB2 and Twist before and after transfection with pcDNA3.1-SATB1 or SATB1-shRNA expression plasmids. These findings were compatible with previous studies and further supported the hypothesis that SATB1 mainly induced EMT through up-regulation of Snail and Slug to repress E-cadherin. However, whether SATB1 directly binds to the MARs of Snail and Slug and also regulates their expression is unknown. Further, whether SATB1 indirectly regulates their expression through other signal pathways to further suppress E-cadherin also remains unknown. Therefore, additional studies were needed to be carried out to clarify the specific mechanisms involved in EMT process. In addition, to define the effects of SATB1 on the biological behavior of bladder cancer cells, a series of cell biological assays, such as cell invasion assays and cell proliferation assays, were performed. Based on our data, we found that ectopic expression of SABT1 increased cell invasive capability and proliferation rate, while SATB1 depletion caused an obvious decrease in cell invasive capacity and proliferation rate in bladder cancer cells. Furthermore, the results indicated that SATB1 overexpression promoted cell cycle progression, but SATB1 depletion inhibited the cell cycle. After SATB1 expression was enhanced, the ratio of cells in G0/G1 phase decreased, and the ratio of cells entering S phase increased significantly, which was important for tumor development and progression. However, there was no difference in the effect of SABT1 deletion and overexpression on cell survival, which was not consistent with a previous study which showed that SATB1inhibited cell apoptotic rates [24,27]. Interestingly, the cell death increased significantly after SATB1 was deleted, so additional experiments will be performed to further explore the mechanism of cell death, such as caspase assays.

Worse clinical outcomes of bladder cancer patients were due to local invasion, tumor diffusion, and distant metastasis [40,41]. Our results were consistent with previous studies on the prognostic value of SATB1 expression in other malignancies [42–44] and thus further provide additional support for the concept that the regulatory activities of SATB1 in cancer preferentially seem to confer a more malignant phenotype [45]. In addition, SATB1 expression was found to be significantly increased in invasive bladder carcinoma compared to non-invasive bladder carcinoma, which further underlined a role for SATB1 in bladder carcinogenesis. The results from this study revealed that elevated expression of SATB1 was significantly associated with age, depth of invasion, TNM stage, lymph node metastasis and distant metastasis but not with the characteristics of gender and tumor differentiation. These results were consistent with Han’s findings in their recent study [27], which provided additional support for the crucial role of SATB1 in the malignant behavior of bladder cancer. Furthermore, the Kaplan-Meier analysis also indicated that those patients with higher SATB1expression levels had shorter overall 5-year survival times, which was in line with previous reports in other human malignancies[9,23,46]. In addition, SATB1 expression was confirmed as a significant and independent prognostic factor for human bladder transitional cell carcinoma by multivariable Cox regression analysis after adjusting for the other factors. On the basis of these findings, we inferred that abnormal expression of SATB1 might contribute to poor survival via involvement with biological aggressiveness, such as deeper tumor invasion, frequent lymph node metastasis and distant metastasis.

In conclusion, we reported for the first time that SATB1 could induce EMT through up-regulation of E-cadherin transcription repressors Snail and Slug, mesenchymal markers vimentin and down-regulation of epithelial markers E-cadherin in an established human bladder cancer cell line. SATB1 was shown to play a crucial role in the development and progression of bladder cancer. Moreover, SATB1 also promoted cell cycle progression, proliferation, migration and increased invasive capability, but had no effect on cell survival. In addition, high SATB1 expression was positively associated with age, depth of invasion, TNM stages, lymph node metastasis and distant metastasis. Furthermore, the patients with high SATB1 expression had reduced 5-year overall survival rate. SATB1 expression is a significant and independent prognostic factor for human bladder transitional cell carcinoma.
